# MicroRNA-325-3p inhibits cell proliferation and induces apoptosis in hepatitis B virus-related hepatocellular carcinoma by down-regulation of aquaporin 5

This article has been retracted.

**DOI:** 10.1186/s11658-019-0137-1

**Published:** 2019-02-12

**Authors:** Zhitao Zhang, Yanzhen Han, Guangxin Sun, Xiaohong Liu, Xiaoyan Jia, Xiangjun Yu

**Affiliations:** 1 General Surgery V Ward, Affiliated Hospital of Hebei Engineering University, Handan, 056002 Hebei Province People’s Republic of China; 2 Clinical Laboratory, Handan Infectious Disease Hospital, Handan, 056002 Hebei Province People’s Republic of China

**Keywords:** Hepatocellular carcinoma, miR-325-3p, Hepatitis B virus, AQP5, Proliferation, Apoptosis

## Abstract

**Background:**

Hepatitis B virus (HBV) infection is acknowledged as the main cause of hepatocellular carcinoma (HCC). Moreover, previous studies have revealed that microRNAs (miRNAs) widely participate in regulation of various cellular processes, such as viral replication. Hence, the purpose of this study was to investigate the roles of aquaporin 5 (AQP5) and miR-325-3p in the proliferation and apoptosis of HBV-related HCC cells.

**Methods:**

AQP5 and miR-325-3p expression in both normal and HBV-HCC tissues or cells (both Huh7–1.3 and HepG2.2.15) was detected using qRT-PCR. AQP5 expression was knocked down in HBV-related Huh7–1.3 and HepG2.2.15 cells using small interfering RNA (siRNA) technology. Down-regulation was confirmed using real-time PCR and Western blot analysis. Effects of AQP5 down-regulation on the proliferation and apoptosis were assessed. Dual luciferase reporter gene assay, Western blot and qRT-PCR were employed to evaluate the effect of miR-325-3p on the luciferase activity and expression of AQP5. Moreover, miR-325-3p mimic-induced changes in cellular proliferation and apoptosis were detected through CCK-8 assay, BrdU assay, flow cytometry analysis and ELISA.

**Results:**

In this study, the expression of AQP5 was up-regulated in human HBV-HCC tissue, Huh7–1.3 and HepG2.2.15 cells. Knockdown of AQP5 significantly inhibited the proliferation and promoted apoptosis of HBV-HCC cells. Next, miR-325-3p was obviously down-regulated in HBV-HCC. In concordance with this, MiR-325-3p directly targeted AQP5, and reduced both mRNA and protein levels of AQP5, which promoted cell proliferation and suppressed cell apoptosis in HCC cells. Overexpression of miR-325-3p dramatically inhibited cell proliferation and induced cell apoptosis.

**Conclusions:**

Our findings clearly demonstrated that introduction of miR-325-3p inhibited proliferation and induced apoptosis of Huh7–1.3 and HepG2.2.15 cells by directly decreasing AQP5 expression, and that silencing AQP5 expression was essential for the pro-apoptotic effect of miR-325-3p overexpression on Huh7–1.3 and HepG2.2.15 cells. It is beneficial to gain insight into the mechanism of HBV infection and pathophysiology of HBV-related HCC.

## Background

Hepatocellular carcinoma (HCC) is the third most common cause of death from cancer worldwide, ranking as the fifth most common cancer in men and the seventh in women [1]. Since HBV is the most frequent underlying cause of HCC, HCC risk is remarkably increased in patients with higher levels of HBV replication [2]. HBx protein, encoded by the HBV X gene, is a multifunctional protein that can modulate cellular transcription, protein degradation, cell cycle, and apoptotic pathways [3]. Many studies have suggested that the HBx protein is important for HBV replication [4–6], and Melegari et al. confirmed that HBx stimulates HBV replication via its transactivation function [7]. Taken together, the evidence shows that HBx activities significantly contribute to the development of HBV-related HCC.

microRNAs (miRNAs), a class of small, non-coding RNAs about 18~25 nucleotides in length, mainly function to negatively regulate gene expression by promoting mRNA degradation or inhibiting mRNA translation through interacting with perfect or imperfect complementary sequences between the miRNA seed and the 3′-untranslated regions (3′-UTR) of its target genes [8]. A growing number of studies have indicated that many miRNAs are involved in the infectious cycle of HBV [9]. For example, miR-101 suppressed HBV replication and expression by targeting forkhead box O1 (FOXO1) [10]; miR-449a facilitated HBV replication by targeting cAMP-responsive element binding protein 5 (CREB5) [11]; transcriptional repression of miR-224 directly targeted the HBV pgRNA and would inhibit HBV replication [12]. Therefore, miRNAs are considered as important regulators in virus infection.

Water channels play a significant role in tumor development, and this finding has been very important for the development of antitumor therapies [13]. Aquaporins (AQPs) are membrane water transport channels that play a role in secretion and absorption in epithelial cells. Some aquaporin subtypes also transport other molecules, such as glycerol and urea. Currently, there are 13 known types of AQPs in mammals, which are mainly divided into 3 categories [14, 15]: 1. classical AQPs, which are primarily water-selective channels, including AQP0, AQP1, AQP2, AQP4, AQP5, AQP6, and AQP8; 2. aquaglyceroporins, including AQP3, AQP7, AQP9, and AQP10, which can also transport glycerol and other small solutes; and 3. non-classical AQPs, including AQP11 and AQP12, which have been localized within cells; however, their selectivity has not been elucidated. In recent years, the roles of AQPs in tumor development have gained increasing attention. Previous studies have shown that AQPs are strongly expressed in tumor cells of different origins and play key roles in tumor biology, including tumor-associated edema, tumor cell migration, tumor proliferation, and tumor angiogenesis [16, 17]. The expression of AQPs in various tumor types differs because of their tissue-specific localization. Recently, the expression of AQP-5 was found to be upregulated in colon cancer tissues. AQP5 expression in colon cancer tissues is related to tumor prognosis, suggesting that AQP5 overexpression is involved in the development of colorectal tumors [18]. AQP5 was reportedly involved in colorectal carcinogenesis [19, 20] and affected the phosphorylation of extracellular signal-regulated kinase-1/2 [21] and p38 MAPK signaling [22] in colorectal cancer cells.

However, the dysregulated level of miR-325-3p in HBV-related HCC has been not reported. In this study, we evaluated the level of miR-325-3p in HBV-related HCC tissues and cell lines, and its effects on proliferation and apoptosis in vitro. We also found that miR-325-3p could negatively regulate the expression of AQP5. It was concluded that miR-325-3p could potentially play a therapeutic role in the near future.

## Materials and methods

### Human tissue samples

Twenty pairs of tumor and adjacent non-cancerous tissues were obtained from patients with HBV-associated HCC at the Affiliated Hospital of Hebei Engineering University (Hebei, China). The tissues were snap-frozen in liquid nitrogen immediately following resection and stored at − 80 °C. Informed consent was obtained from all subjects (patient or the patient’s family). The study was approved by the Ethics Committee of the Affiliated Hospital of Hebei Engineering University (HEU2017081121) and it complies with the guidelines and principles of the Declaration of Helsinki.

### Cell culture

Hepatoma cell lines HepG2, HepG2.2.15, and Huh7 cells purchased from American Type Culture Collection (ATCC) were maintained in Dulbecco’s modified Eagle’s medium (DMEM; Gibco, USA) supplemented with 10% fetal bovine serum (FBS; Hyclone, USA), and 100 μg/ml streptomycin solution and 100 U/ml penicillin at 37 °C in a humidified incubator with 5% CO_2_. The HepG2.2.15 cells were established by transfecting the HBV genome into HepG2 cells and selecting with G418. Huh7–1.3 cells were established by transfection with recombinant pcDNA 3.0–1.3 mer which contained the 1.3 mer fragment of HBV genomic DNA with FuGENE HD Transfection Reagent (Promega, USA) in accordance with the manufacturer’s instructions.

### Transient transfection

The miR-325-3p mimic, miR-negative control of mimic (miR-NC), pcDNA-AQP5 and pcDNA3.1 vectors were synthesized and purified by Gene-Pharma (Shanghai, China). Huh7–1.3 and HepG2.2.15 cells were transfected with 50 nM miR-325-3p mimic and miR-NC using Lipofectamine 3000 reagent (Invitrogen, Carlsbad, CA, USA) following the manufacturer’s protocols. Total RNA and protein were collected 48 h after transfection.

### RNA extraction and quantitative real time-polymerase chain reaction (qRT-PCR)

Total RNA was extracted using the TRIzol reagent (Invitrogen, USA), according to the manufacturer’s instructions. cDNA was synthesized from 2 μg of total RNA using a PrimeScript RT reagent kit (Takara, Tokyo, Japan), according to the manufacturer’s protocol. The PCR reaction was performed in a volume of 20 μl. The PCR program was as follows: 95 °C for 1 min; 40 cycles of 95 °C for 15 s, 60 °C for 20 s, and 72 °C for 40 s; and 72 °C for 7 min. The relative expression of each gene was calculated using the 2^ΔΔCt^ method.

### Cell viability

For estimating cell viability, a Cell Counting Kit-8 (CCK-8) (Thermo Fisher Scientific, Carlsbad, CA, USA) assay was performed. Huh7–1.3 and HepG2.2.15 cells were seeded in 96-well culture plates at 2 × 10^4^ cells per well. After 24 h, the cells were transfected with miR-325-3p mimic and miR-NC for 48 h. Then, 10 μl of CCK-8 reagents were separately added into each well before transfection and after transfection. The cell viability rates were shown by the OD value at 450 nm via a microplate reader (Bio-Rad, USA).

### Cell proliferation assay

To explore the effect of miR-325-3p on proliferation of Huh7–1.3 and HepG2.2.15 cells, 2 × 10^4^ cells were seeded in a 96-well plate and allowed to grow overnight in complete medium. The medium was removed, and then cells were transfected with miR-325-3p mimic or miR-NC for 48 h at 37 °C. The Cell Proliferation ELISA-BrdU (colorimetric) Kit (Roche, Inc., Switzerland) was used to detect the cell proliferation according to the manufacturer’s protocols.

### Flow cytometry assay for apoptosis

Apoptosis was detected using the Annexin V-FITC/PI Apoptosis Detection Kit according to the manufacturer’s instructions. Each well of the 6-well plate was inoculated with 10^5^ cells. The medium was discarded after 24 h of incubation, and the wells were washed once with PBS, followed by transfection and a second 24-h incubation. The cells were trypsinized and centrifuged, and then stained with Annexin V and propidium iodide in the dark for 15 min. The percentage of apoptotic cells in each sample was determined by flow cytometry.

### Detection of apoptosis

According to a previous study [23], apoptosis was determined using the Cell Death ELISA Detection Kit (Roche), which measures cytoplasmic DNA-histone complexes generated during apoptotic DNA fragmentation. Cell apoptosis detection was performed under the manufacturer’s instructions and monitored spectrometrically at 405 nm.

### Caspase-3 activity assay

A caspase-3 fluorescent assay kit (Nanjing KeyGEN Biotech. CO., LTD, China) was used to detect caspase activity according to a previous study (18). Briefly, after treatment, cells were lysed in the lysis buffer and centrifuged at 10,000×g for 1 min, and then the supernatants were collected. Equal amounts of protein samples were reacted with the synthetic fluorescent substrates at 37 °C for 1.5 h and the reactions were read at 405 nm in a microplate reader (Bio-Rad). Fold increases in caspase-3 activity were determined with values obtained from the treatment samples divided by those from the controls.

### Western blot analysis

After transfection with miR-325-3p mimic and miR-NC for 48 h, Huh7–1.3 and HepG2.2.15 cells were washed twice in cold PBS, and then lysed in RIPA lysis buffer (Beyotime Institute of Biotechnology, Jiangsu, China) with protease inhibitor cocktail (Merck, Germany) to extract protein. The protein concentration of cell lysates was quantified using the BCA Kit (Beyotime Institute of Biotechnology). The proteins were separated by 10% SDS-PAGE and blotted onto a nitrocellulose membrane by semi-dry transfer. Next, the membrane was blocked by immersion in Tris-buffered saline with Tween 20 (TBST) containing 5% skim milk and overnight incubation with the primary antibody against AQP5 (Abcam, ab92320) at 4 °C. On the following day, the membrane was incubated with the secondary antibody conjugated to horseradish peroxidase (1:2000; Santa Cruz) at 25 °C for 2 h, and then an enhanced chemiluminescence kit (Amersham Pharmacia Biotech, Amersham, UK) was used for staining. The membrane was photographed, and the results were analyzed.

### Extraction and quantification of HBV cccDNA

The samples were treated with 10 μg DNase I for 16 h at 37 °C. 100 μl of lysis buffer (20 mM Tris-HCl, 20 mM EDTA, 50 mM NaCl and 0.5% SDS) containing 50 μg proteinase K were added. After incubation at 65 °C for 3 h, viral DNA was isolated by phenol/chloroform extraction and ethanol precipitation. The DNA pellet was rinsed with 70% ethanol and re-suspended in 10 μl of ddH_2_O. The cccDNA was later subjected to real-time-PCR using SYBR Green Real-time PCR Master Mix (Roche, Germany) and cccDNA-specific primers: 5′-TGCACTTCGCTTCACCT (forward) and 5′-AGGGGCATTTGGTGGTC (reverse). PCR was performed using the ABI PRISM 7500 Sequence Detection System (Applied Biosystems, USA). The average threshold cycle values were used to determine the concentration of HBV DNA. The inhibitory rate was calculated according to the formula: inhibitory rate (%) = (Ccontrol-Ctested)/Ccontrol× 100%.

### Detection of HBsAg and HBeAg

The collected cellular supernatant was used to detect the level of HBV surface antigen (HBsAg) and antigen (HBeAg) with commercially available ELISA kits (InTec, China) in line with the instructions of the supplier. A standard curve was drawn with the optical density (OD) values on the ordinate axis and standard concentrations on the abscissa axis. The corresponding concentrations were found on the standard curve with the OD values. Inhibitory rates were calculated according to the formula: inhibitory rate (%) = (Ccontrol-Ctested)/Ccontrol× 100%. Each experiment was repeated three times to obtain the mean values.

### Luciferase reporter assay

The amplified human 3′-UTR segments of the AQP5 gene (containing the predicted miR-325-3p binding site) were inserted into psiCHECK-2 vectors (Promega, USA) containing Renilla luciferase (Promega, USA) to generate the wild-type plasmid (AQP5 3′-UTR WT) or mutant plasmid (AQP5 3′-UTR MUT) constructs. All constructs were further verified by sequencing. For luciferase assays, 293 T cells were seeded in 96-well plates and co-transfected with the recombinant vectors along with control psiCHECK-2 plasmid, miR-325-3p mimics or negative control (NC) plasmid using Lipofectamine 2000 reagent. The cells were collected and analyzed by applying the Dual-Luciferase Reporter Assay System (Promega, USA) after 48 h. The luciferase activity values were normalized relative to that of the Renilla luciferase internal control. Each experiment was repeated three times in duplicate.

### Statistical analysis

All statistical analyses were performed using GraphPad Prism 5.0 (GraphPad Software, Inc., USA). Data from each group were expressed as mean ± standard error of the mean (S.E.M.) and statistically analyzed by Student’s t test. Differences were considered statistically significant at a *p* value of < 0.05.

## Results

### Expression of AQP5 and its effects on cell proliferation and apoptosis of HBV-HCC cells

It has been reported that AQPs (such as AQP1, AQP3, AQP4, AQP5 and AQP6) are closely associated with cancers. However, it is still unknown which ones play a critical role in HBV-HCC. In this study, we detected expression of AQP1, AQP3, AQP4, AQP5 and AQP6 genes in HBV-HCC tissues. The results showed that the mRNA level of AQP5 was the highest in HBV-HCC tissues among these five AQP genes compared with the adjacent tissues (Fig. 1a). To confirm the tendency of the AQP5 level to increase, we then determined the expression of AQP5 in Huh7 and Huh7–1.3, and HepG2 and HepG2.2.15 by qRT-PCR and Western blot, respectively. The results showed that AQP5 was also obviously higher in Huh7–1.3 and HepG2.2.15 than in Huh7 and HepG2, respectively (Fig. 1b).

**Fig. 1:** Expression of AQP5 and its effects on cell proliferation and apoptosis of HBV-HCC cells. **a** mRNA and protein expression of AQP1, AQP3, AQP4, AQP5 and AQP6 in normal liver tissues (*n* = 20) and HBV-HCC tissues (*n* = 20) was detected by qRT-PCR. **b** mRNA expression of AQP5 in HepG2, HepG2.2.15, Huh7 and Huh7–1.3 cells. Cell proliferation was assessed by CCK-8 assay (**c**) and BrdU-ELISA assay (**d**). Cell apoptosis was measured by flow cytometric analysis of cells labeled with Annexin-V/PI double staining (**e**) and nucleosomal degradation using Roche’s cell death ELISA detection kit (**f**). The data shown are mean ± SEM, *n* = 4. *P < 0.05, ***p < 0.001 vs. normal tissues; ^##^*p* < 0.01 vs. HepG2, Huh7 or si-NC

To study the role of AQP5 in Huh7–1.3 and HepG2.2.15 cells, cell proliferation and apoptosis were estimated after transfection with si-NC or si-AQP5 for 48 h. The CCK-8 and BrdU assays indicated that knockdown of AQP5 significantly suppressed the proliferation of Huh7–1.3 and HepG2.2.15 cells (Fig. 1c, d). Furthermore, knockdown of AQP5 promoted cell apoptosis of Huh7–1.3 and HepG2.2.15 cells (Fig. 1e, f).

### AQP5 was identified as one of the direct targets of miR-325-3p

Subsequently, we predicted that miR-325-3p could directly target AQP5 by bioinformatics. Our results showed that the miR-325-3p level was significantly reduced in HBV-HCC tissues and cells (Fig. 2a, b). Taken together, these data suggested that the decreased miR-325-3p expression was closely related to HBV-HCC. To study whether the AQP5 expression was closely associated with miR-325-3p in HBV-HCC tissues or not, the Pearson’s correlation analysis revealed a significant inverse correlation between AQP5 and miR-325-3p in HBV-HCC tissues (Fig. 2c). To identify putative targets of miR-325-3p, the online database TargetScan 7.2 was used in this study. The AQP5 was simultaneously predicted to have a complementary site at the 3′-UTR with miR-325-3p, and preliminarily recognized as a putative target of miR-325-3p. The prediction results are listed in Fig. 2d.

**Fig. 2:** AQP5 was a direct target of miR-325-3p. **a** Levels of miR-325-3p in normal liver tissues (*n* = 20) and HBV-HCC tissues (*n* = 20) were detected by qRT-PCR. **b** Levels of miR-325-3p in HepG2, HepG2.2.15, Huh7 and Huh7–1.3 cells. **c** Pearson’s correlation analysis of the relative expression levels of miR-325-3p and the relative AQP5 mRNA levels in HBV-HCC tissues. **d** Schematic representation of AQP5 3′-UTRs showing putative miRNA target site. **e** mRNA expression of AQP5 was determined by qRT-PCR in Huh7–1.3 and HepG2.2.15 cells transfected with miR-325-3p mimic or miR-NC. **f** Protein expression of AQP5 was determined by Western blot in Huh7–1.3 and HepG2.2.15 cells transfected with miR-325-3p mimic or miR-NC. **g** Analysis of the relative luciferase activities of AQP5-WT and AQP5-MUT in Huh7–1.3 and HepG2.2.15 cells. All data are presented as mean ± SEM, *n* = 6. ***P < 0.001 vs. normal tissues; ^##^*p* < 0.01, ^###^*p* < 0.001 vs. HepG2, Huh7 or miR-NC

Referring to the decreased level of miR-325-3p and increased expression of AQP5 in HBV-HCC tissues and cells, we carried out qRT-PCR and Western blotting to determine the effect of miR-325-3p overexpression on target AQP5. The qRT-PCR analysis showed that the expression of AQP5 was obviously decreased after overexpression of miR-325-3p at the mRNA level (Fig. 2e). The Western blotting analysis revealed that the expression of AQP5 was also significantly lowered at protein levels in Huh7–1.3 and HepG2.2.15 cells transfected with miR-325-3p mimic compared to the miR-NC group (Fig. 2f). To further demonstrate the interaction of miR-325-3p and 3′-UTR region of AQP5, we performed the dual luciferase reporter assays. After co-transfection of miR-325-3p mimic and pGL3-AQP5, the luciferase activity was dramatically reduced compared to the miR-NC group (Fig. 2g). Altogether, these results demonstrated that AQP5 was indeed one direct downstream target of miR-325-3p in HBV-HCC.

### MiR-325-3p inhibited secretion of HBV and replication of HBV-DNA

The qRT-PCR analysis showed that the miR-325-3p level was significantly increased in the miR-325-3p mimic group compared to the miR-NC group in Huh7–1.3 and HepG2.2.15 cells (Fig. 3a). HBeAg positivity and HBsAg positivity were both considered as evidence of HBV infection. In this study, we found that the concentrations of HBeAg and HBsAg were increased in Huh7–1.3 and HepG2.2.15 cells as compared to Huh7 and HepG2 cells (Fig. 3b, c). Moreover, the levels of released nuclear HBV cccDNA were also elevated in Huh7–1.3 and HepG2.2.15 cells relative to Huh7 and HepG2 cells (Fig. 3d). Subsequently, the effect of miR-325-3p on HBV antigen levels and HBV replication in Huh7–1.3 and HepG2.2.15 cells was further investigated. ELISA and PCR experiments revealed strong reductions in HBeAg (Fig. 3b), HBsAg (Fig. 3c) and cccDNA levels (Fig. 3d), indicating that miR-325-3p might inhibit HBV antigen secretions and viral replication.

**Fig. 3:** miR-325-3p inhibited HBV antigen secretion and viral replication. Huh7–1.3 and HepG2.2.15 cells were transfected with miR-325-3p mimic or miR-NC for 48 h. (A) Levels of miR-325-3p in Huh7–1.3 and HepG2.2.15 cells were determined by qRT-PCR. (B) Culture medium from each group was collected and detected for levels of HBeAg by ELISA. (C) Culture medium from each group was harvested and measured for levels of HBsAg by ELISA. (D) Levels of released of nuclear HBV cccDNA were determined by quantitative PCR in each group. All data are presented as mean ± SEM, *n* = 6. ^#^*p* < 0.05, ^##^*p* < 0.01, ^###^*p* < 0.001 vs. miR-NC

### MiR-325-3p inhibited proliferation and induced apoptosis

To preliminarily determine the biological effects of miR-325-3p on cell viabilities, proliferation and apoptosis, we performed CCK-8, BrdU and ELISA assays after transfection with miR-325-3p mimic in both Huh7–1.3 and HepG2.2.15 cells. The CCK-8 and BrdU assays revealed that overexpression of miR-325-3p significantly inhibited the proliferation of Huh7–1.3 and HepG2.2.15 cells (Fig. 4a, b). For further study, ELISA assays demonstrated that miR-325-3p dramatically induced cell apoptosis of Huh7–1.3 and HepG2.2.15 cells (Fig. 4c). Finally, to confirm the above apoptosis results, we detected the caspase 3 activity. After transfection with miR-325-3p mimic, the activity of caspase 3 was significantly increased (Fig. 4d). Altogether, increased miR-325-3p expression significantly inhibited the proliferation and induced apoptosis of Huh7–1.3 and HepG2.2.15 cells.

**Fig. 4:** Effects of miR-325-3p on cell proliferation and apoptosis in Huh7–1.3 and HepG2.2.15 cells. Huh7–1.3 and HepG2.2.15 cells were transfected with miR-325-3p mimic or miR-NC for 48 h. Cell proliferation was assessed by CCK-8 assay (**a**) and BrdU-ELISA assay (**b**). (**c**) Cell apoptosis was measured by nucleosomal degradation using Roche’s cell death ELISA detection kit. **d** Activities of caspase-3 were determined by caspase-3 activity detection assay. All data are presented as mean ± SEM, *n* = 6. ^#^*p* < 0.05, ^##^*p* < 0.01 vs. miR-NC

### Introduction of AQP5 reversed the effects of miR-325-3p mimic on proliferation and apoptosis of Huh7–1.3 and HepG2.2.15 cells

To determine whether miR-325-3p overexpression protected HCC cells from HBV-induced apoptosis in an AQP5-dependent manner, we cotransfected Huh7–1.3 and HepG2.2.15 cells with miR-325-3p mimic and pcDNA-AQP5. We found that the expression of AQP5 was dramatically increased after transfection with miR-325-3p mimic and pcDNA-AQP5 compared with miR-325-3p mimic and pcDNA3.1 in Huh7–1.3 and HepG2.2.15 cells (Fig. 5a, b). Analysis by CCK-8 and BrdU assays indicated that up-regulation of AQP5 in cells transfected with the miR-325-3p mimic increased the proliferation of Huh7–1.3 and HepG2.2.15 cells transfected with miR-325-3p mimic only (Fig. 5c, d). Moreover, our results also showed that overexpression of AQP5 could reverse the pro-apoptotic effect of miR-325-3p mimic on Huh7–1.3 and HepG2.2.15 cells (Fig. 5e, f). Our findings clearly demonstrated that introduction of miR-325-3p inhibited proliferation and induced apoptosis of Huh7–1.3 and HepG2.2.15 cells by directly decreasing AQP5 expression, and that silencing AQP5 expression was essential for the pro-apoptotic effect of miR-325-3p overexpression on Huh7–1.3 and HepG2.2.15 cells.

**Fig. 5:** Effects of AQP5 overexpression on cell proliferation and apoptosis in Huh7–1.3 and HepG2.2.15 cells transfected with miR-325-3p mimic. Huh7–1.3 and HepG2.2.15 cells were transfected with miR-325-3p mimic and pcDNA-AQP5 or pcDNA3.1. Expression of AQP5 was detected by Western blot (**a**) and qRT-PCR (**b**). Cell proliferation was assessed by CCK-8 assay (**c**) and BrdU-ELISA assay (**d**). **e** Cell apoptosis was measured by nucleosomal degradation using Roche’s cell death ELISA detection kit. **f** The activities of caspase-3 were determined by caspase-3 activity detection assay. All data are presented as mean ± SEM, *n* = 6. ^#^*p* < 0.05, ^##^*p* < 0.01, ^###^*p* < 0.001 vs. miR-325-3p mimic + pcDNA3.1

## Discussion

AQPs are specific channels for highly efficient and selective transport of water molecules and are widely present in the cell membranes of prokaryotes and eukaryotes [24]. Tumor development involves a loss of the normal regulation of cell growth at the genetic level due to various tumorigenic factors. Tumors rely on various metabolic processes involving water molecules, and AQPs can rapidly and specifically transport water molecules [25]. AQP1–12 is widely expressed in the brain, skin, fat, liver, kidney, pancreas, muscle, ovary, testis, spleen, lung, and tissues where body fluid absorption and secretion occur [26]. AQPs are also involved in the reabsorption of water in the kidneys, gland secretion, intestinal lipid absorption, and function at the blood-air barrier, blood-brain barrier, and in cerebrospinal fluid formation [26]. Additionally, AQPs are involved in the stress response, tissue injury, infection, and tumor formation [25]. Different AQPs are expressed in different types of tumors because of their tissue-specific localization, for example, AQP1 expression is often associated with brain tumors [27]. In a study of AQP3-null mice, deletion of the AQP3 gene induced resistance to carcinogen-induced skin tumors [28]. In addition, AQP3-facilitated glycerol transport contributes to ATP production during cell proliferation and tumorigenesis [28]. High expression levels of AQP5 in breast [29], stomach [30], liver [31], lung [32], and cervical [33] cancers are associated with poor prognosis.

AQPs play a key role in maintaining water balance and regulating various physiological and pathological processes [34]. AQP5 is a 21–24-kDa protein that was initially thought to be the major structural protein of caveolae in cell membranes and was shown to be a key molecule in oncogenic transformation and malignant progression [35, 36]. Previous studies have shown that high AQP5 expression can promote cell proliferation, inhibit cell apoptosis, reset the cell cycle, and promote epithelial-mesenchymal transition and cell migration [37]. Our preliminary study indicated that the AQP5 expression was significantly increased in HBV-HCC tissues. In further study, we found out that HBV-related Huh7–1.3 and HepG2.2.15 cells exhibit higher AQP5 mRNA and protein expression levels than in Huh7 and HepG2 cells, suggesting that AQP5 overexpression may be regulated by HBV infection at the transcriptional level. To uncover the role of AQP5 in the development of HBV-related HCC, we employed a loss-of-function approach to assess the effects of AQP5 down-regulation on the growth and survival of Huh7–1.3 and HepG2.2.15 cells. SiRNA-mediated down-regulation of AQP5 significantly inhibited cell proliferation, indicating that AQP5 is required for HCC cell growth. In addition to inhibition of cell proliferation, AQP5 down-regulation was also found to promote apoptosis in Huh7–1.3 and HepG2.2.15 cells. In concordance with annexin-V/PI double labeling analysis, the activity of caspase-3 was increased in AQP5 transfected cells compared to the control cells. Caspase-3 is a crucial executioner of cell apoptosis in caspase signaling [38].

It is well known that miRNAs act as key factors in several biological processes, such as cell proliferation, differentiation and apoptosis [39]. Moreover, evidence is emerging that miRNAs are key mediators in the replication and propagation of viruses [40]. For example, miR-23b detected in Enterovirus 71 (EV71)-infected cells could inhibit virus replication by targeting the EV71 VP1 RNA coding region [41]; miR-548 g-3p suppressed the recruitment of the viral RNA-dependent RNA polymerase (NS5) to the viral genome, which ultimately resulted in a blockade of viral replication via targeting the stem loop A promoter element of Dengue virus (DENV) 5′-UTR [42]. In the present study, we found that miR-325-3p overexpression by transfection of a miR-325-3p mimic into Huh7–1.3 and HepG2.2.15 cells inhibited HBV antigen secretions, including HBeAg and HBsAg, and viral cccDNA replication. The levels of released of HBeAg and HBsAg are commonly used to analyze the conditions of HBV replication [43]. Therefore, our results suggest that miR-325-3p might repress HBV replication. Subsequently, based on the inverse expression of miR-325-3p and AQP5, a dual-luciferase reporter assay was used to identify the interaction between miR-325-3p and AQP5, and the data revealed that miR-325-3p could directly target 3′-UTR of AQP5. Additionally, miR-325-3p mimic transfection in Huh7–1.3 and HepG2.2.15 cells further verified that overexpression of miR-325-3p significantly inhibited cell proliferation and promoted cell apoptosis. Finally, introduction of AQP5 reversed the effects of miR-325-3p mimic on cell proliferation and apoptosis of Huh7–1.3 and HepG2.2.15 cells.

## Conclusions

Our results showed that miR-325-3p was down-regulated in HBV-HCC tissues and cells. miR-325-3p inhibited cell proliferation and induced apoptosis through the suppression of AQP5, functioning as a tumor suppressor. Moreover, the down-regulation of miR-325-3p after HBV infection led to increasing expression of one target AQP5, which might play important roles in chronic HBV infection and HCC development. In conclusion, our study provided a novel miRNA which is beneficial to gain insight into the mechanism of and pathophysiology of HBV-related HCC.

## Abbreviations

AQP: Aquaporins
HBV: Hepatitis B virus
HCC: Hepatocellular carcinoma
miRNA: microRNA
qRT-PCR: quantitative real-time-polymerase chain reaction

## References

[1] Ferlay J, Shin HR, Bray F, Forman D, Mathers C, Parkin DM (2010). Estimates of worldwide burden of cancer in 2008: GLOBOCAN 2008. International journal of cancer. Int J Cancer.

[2] El-Serag HB, Rudolph KL (2007). Hepatocellular carcinoma: epidemiology and molecular carcinogenesis. Gastroenterology.

[3] Kew MC (2011). Hepatitis B virus x protein in the pathogenesis of hepatitis B virus-induced hepatocellular carcinoma. J Gastroenterol Hepatol.

[4] Bouchard MJ, Wang LH, Schneider RJ (2001). Calcium signaling by HBx protein in hepatitis B virus DNA replication. Science.

[5] Keasler VV, Hodgson AJ, Madden CR, Slagle BL (2007). Enhancement of hepatitis B virus replication by the regulatory X protein in vitro and in vivo. J Virol.

[6] Tsuge M, Hiraga N, Akiyama R, Tanaka S, Matsushita M, Mitsui F, Abe H, Kitamura S, Hatakeyama T, Kimura T, Miki D, Mori N, Imamura M, Takahashi S, Hayes CN, Chayama K (2010). HBx protein is indispensable for development of viraemia in human hepatocyte chimeric mice. J Gen Viroly.

[7] Melegari M, Wolf SK, Schneider RJ (2005). Hepatitis B virus DNA replication is coordinated by core protein serine phosphorylation and HBx expression. J Virol.

[8] Liu X, Fortin K, Mourelatos Z (2008). MicroRNAs: biogenesis and molecular functions. Brain Pathol.

[9] Deng W, Lu M (2016). The role of microRNAs in hepatocyte metabolism and hepatitis B virus replication. Virol Sin.

[10] Wang Y, Tian H (2017). miR-101 suppresses HBV replication and expression by targeting FOXO1 in hepatoma carcinoma cell lines. Biochem Biophys Res Commun.

[11] Zhang X, Liu H, Xie Z, Deng W, Wu C, Qin B, Hou J, Lu M (2016). Epigenetically regulated miR-449a enhances hepatitis B virus replication by targeting cAMP-responsive element binding protein 5 and modulating hepatocytes phenotype. Sci Rep.

[12] Guerrieri F, Belloni L, D’Andrea D, Pediconi N, Le Pera L, Testoni B, Scisciani C, Floriot O, Zoulim F, Tramontano A, Levrero M (2017). Genome-wide identification of direct HBx genomic targets. BMC Genomics.

[13] Sekine S, Shimada Y, Nagata T, Moriyama M, Omura T, Watanabe T, Hori R, Yoshioka I, Okumura T, Sawada S, Fukuoka J, Tsukada K (2012). Prognostic significance of aquaporins in human biliary tract carcinoma. Oncol Rep.

[14] Ishibashi K, Tanaka Y, Morishita Y (2014). The role of mammalian superaquaporins inside the cell. Biochim Biophys Acta.

[15] Benga G (2012). On the definition, nomenclature and classification of water channel proteins (aquaporins and relatives). Mol Asp Med.

[16] Verkman AS, Hara-Chikuma M, Papadopoulos MC (2008). Aquaporins--new players in cancer biology. J Mol Med (Berl).

[17] Papadopoulos MC, Saadoun S (2015). Key roles of aquaporins in tumor biology. Biochim Biophys Acta.

[18] Shan T, Cui X, Li W, Lin W, Li Y (2014). AQP5: a novel biomarker that predicts poor clinical outcome in colorectal cancer. Oncol Rep.

[19] Kang SK, Chae YK, Woo J, Kim MS, Park JC, Lee J, Soria JC, Jang SJ, Sidransky D, Moon C (2008). Role of human aquaporin 5 in colorectal carcinogenesis. Am J Pathol.

[20] Moon C, Soria JC, Jang SJ, Lee J, Obaidul Hoque M, Sibony M, Trink B, Chang YS, Sidransky D, Mao L (2003). Involvement of aquaporins in colorectal carcinogenesis. Oncogene.

[21] Woo J, Lee J, Chae YK, Kim MS, Baek JH, Park JC, Park MJ, Smith IM, Trink B, Ratovitski E, Lee T, Park B, Jang SJ, Soria JC, Califano JA, Sidransky D, Moon C (2008). Overexpression of AQP5, a putative oncogene, promotes cell growth and transformation. Cancer Lett.

[22] Shi X, Wu S, Yang Y, Tang L, Wang Y, Dong J, Lu B, Jiang G, Zhao W (2014). AQP5 silencing sup- presses p38 MAPK signaling and improves drug resistance in colon cancer cells. Tumour Biol.

[23] Zhao Z, Li C, Xi H, Gao Y, Xu D (2015). Curcumin induces apoptosis in pancreatic cancer cells through induction of forkhead box o1 (FOXO1) and inhibition of PI3K/Akt pathway. Mol Med Rep.

[24] Abascal F, Irisarri I, Zardoya R (2014). Diversity and evolution of membrane intrinsic proteins. Biochim Biophys Acta.

[25] Ribatti D, Ranieri G, Annese T, Nico B (2014). Aquaporins in cancer. Biochim Biophys Acta.

[26] Ishibashi K, Hara S, Kondo S (2009). Aquaporin water channels in mammals. Clin Exp Nephrol.

[27] Wang D, Owler BK (2011). Expression of AQP1 and AQP4 in paediatric brain tumours. J Clin Neurosci.

[28] Hara-Chikuma M, Verkman AS (2008). Prevention of skin tumorigenesis and impairment of epidermal cell proliferation by targeted aquaporin-3 gene disruption. Mol Cell Biol.

[29] Lee SJ, Chae YS, Kim JG, Kim WW, Jung JH, Park HY, Jeong JY, Park JY, Jung HJ, Kwon TH (2014). AQP5 expression predicts survival in patients with early breast cancer. Ann Surg Oncol.

[30] Shen L, Zhu Z, Huang Y, Shu Y, Sun M, Xu H, Zhang G, Guo R, Wei W, Wu W (2010). Expression profile of multiple aquaporins in human gastric carcinoma and its clinical significance. Biomed Pharmacother.

[31] Guo X, Sun T, Yang M, Li Z, Li Z, Gao Y (2013). Prognostic value of combined aquaporin 3 and aquaporin 5 overexpression in hepatocellular carcinoma. Biomed Res Int.

[32] Chae YK, Woo J, Kim MJ, Kang SK, Kim MS, Lee J, Lee SK, Gong G, Kim YH, Soria JC, Jang SJ, Sidransky D, Moon C (2008). Expression of aquaporin 5 (AQP5) promotes tumor invasion in human non small cell lung cancer. PLoS One.

[33] Zhang T, Zhao C, Chen D, Zhou Z (2012). Overexpression of AQP5 in cervical cancer: correlation with clinicopathological features and prognosis. Med Oncol.

[34] McCoy E, Sontheimer H (2007). Expression and function of water channels (aquaporins) in migrating malignant astrocytes. Glia.

[35] Zhang Z, Chen Z, Song Y, Zhang P, Hu J, Bai C (2010). Expression of aquaporin 5 increases proliferation and metastasis potential of lung cancer. J Pathol.

[36] Jung HJ, Park JY, Jeon HS, Kwon TH (2011). Aquaporin-5: a marker protein for proliferation and migration of human breast cancer cells. PLoS One.

[37] Direito I, Madeira A, Brito MA, Soveral G (2016). Aquaporin-5: from structure to function and dysfunction in cancer. Cell Mol Life Sci.

[38] Budayeva HG, Rowland EA, Cristea IM (2015). Intricate roles of mammalian sirtuins in defense against viral pathogens. J Virol.

[39] Davis-Dusenbery BN, Hata A (2010). Mechanisms of control of microRNA biogenesis. J Biochem.

[40] Drury RE, O’Connor D, Pollard AJ (2017). The clinical application of MicroRNAs in infectious disease. Front Immunol.

[41] Wen BP, Dai HJ, Yang YH, Zhuang Y, Sheng R (2013). MicroRNA-23b inhibits enterovirus 71 replication through downregulation of EV71 VPl protein. Intervirology.

[42] Wen W, He Z, Jing Q, Hu Y, Lin C, Zhou R, Wang X, Su Y, Yuan J, Chen Z, Yuan J, Wu J, Li J, Zhu X, Li M (2015). Cellular microRNA-miR-548g-3p modulates the replication of dengue virus. J Inf Secur.

[43] Wei ZQ, Zhang YH, Ke CZ, Chen HX, Ren P, He YL, Hu P, Ma DQ, Luo J, Meng ZJ (2017). Curcumin inhibits hepatitis B virus infection by down-regulating cccDNA-bound histone acetylation. World J Gastroenterol.

